This article has been retracted.

# The Mongolian Vowel Acoustic Model Based on the Clustering Algorithm

**DOI:** 10.1155/2022/1917350

**Published:** 2022-10-15

**Authors:** Wujisguleng

**Affiliations:** Mongolian Studies College, Inner Mongolia Minzu University, Inner Mongolia, Tongliao 028000, China

## Abstract

In order to solve the problem of vowel acoustic modeling in the Mongolian language and provide more scientific core technical support for speech recognition system, a vowel acoustic model based on the clustering algorithm and speech recognition technology was proposed. The language vowel recognition system and Mongolian speech recognition system are constructed, the Mongolian vowel acoustic database is mainly designed, and the number of vowel samples is constantly increased to ensure the acoustic and linguistic phenomena that may be encountered in the Mongolian vowel database. At the same time, classification modeling and context modeling are used to improve the accuracy of the acoustic model. Through experiments, it is found that the experimental results of sparse tritones show that the model has the highest recognition accuracy of 45% for sentences and 86% for words, which is more than 2% higher than before, providing some technical support for Mongolian learning and pronunciation.

## 1. Introduction

Speech recognition is to convert human language information into corresponding text or command through the recognition and understanding of speech with the help of machine learning technology, which is also an important topic in the field of artificial intelligence research in recent years. The development of speech recognition technology is bound to have a profound impact on the future human-computer interface [1]. In the research process of speech recognition, it is the most challenging problem for specific people; large vocabulary and continuous speech recognition are the most difficult research topic for vowel recognition of minority languages. The object of this study is the Mongolian language. With the deepening of the international information wave, the Mongolian autonomous region is rapidly entering the information society; in this process, Mongolian has gradually become a relatively influential language in the world, which is why it is of great practical significance to construct the vowel acoustic model of the Mongolian language.

The 1950s can be said to be the initial stage of the exploration of speech recognition technology, during which researchers mainly from the angle of acoustic phonetics sought to solve the problem of speech recognition. A milestone in the development of automatic speech recognition devices is the Audrey system developed by some scholars. The speech recognition system can recognize the pronunciation of isolated words in English by specific speakers based on the variation information of vowel formant frequency extracted by analog components. Other research achievements of this period include the following: some scholars developed a phoneme recognizer for recognizing four vowels and nine consonants [2]. The novelty of this research lies in the introduction of statistical grammar in speech recognition to improve the accuracy of phoneme recognition. Some scholars have developed a vowel recognizer that can recognize ten vowels in a specific context. Its progress is that the system is targeted at the nonspecific pronunciation network.

## 2. Related Works

With the advent of the new century, the research on speech recognition has taken on a new look. DARPA continues to focus on speech recognition research, launching global autonomous language development projects in 2002, 2011, and 2012 to use computer software to retrieve, analyze, and translate vast volumes of multilingual speech and text, so as to mainly solve the problems of the robust automatic speech tagging project focused on speech recognition, speaker recognition, and language recognition in noisy environments and to design a multilingual translation project to accurately translate narrow Mandarin and multiple Arabic dialects from a variety of media into English [3]. While integrating increasingly sophisticated speech recognition technologies, these projects have put higher demands on the technology itself, and more emphasis on speech recognition and other cutting-edge technology organic integration and comprehensive application is increased. The discriminative training technique of the acoustic model in HMM framework has been developed in depth. For example, the minimum word/phoneme error discriminative training criterion was proposed at the same time; a new acoustic model that jumped out of the HMM framework was also explored and deep learning became a new research frontier in the field of machine learning and artificial intelligence. Specifically, the application of deep learning in speech recognition. With the improvement of computer hardware performance and the progress of machine learning algorithms [4]. The idea of using the neural network to replace the gaussian mixture model in the hidden Markov model proposed in the 1990s has gained attention again, and the theory and method of using the multilayer deep neural network to replace GMM have achieved great success in practice, which has become a new milestone in the field of speech recognition. New extension applications based on simple speech recognition, such as speech retrieval and multimodal speech recognition, have gradually emerged and become an important research field [5].

## 3. The Clustering Analysis Algorithm

The clustering algorithm is an important branch of machine learning and generally adopts unsupervised learning. Using the clustering analysis algorithm, the data in the database can be divided into several categories. The distance between individuals in the same category is small, so the objects in the cluster have high similarity. However, the distance between individuals in different categories is relatively large, with great differences [6]. The clustering model can be described as follows:

*n* data objects in *m* dimensional space *R*^*m*^ are divided, and the vector with the smallest distance from the cluster center is assigned to the corresponding K-means cluster. In cluster analysis, *j* is the number of attributes of the cluster sample, *n* is the number of samples, and *k* is the number of classifications preset by the user. The mathematical model is as follows:

for vectors *X*_*i*_、*X*_*j*_ of *m* dimensional space *R*^*m*^, the following formulas are considered:

(1) $$\begin{array}{c} X_{i}=\left\{X_{i1},X_{i2},X_{im}\right\}\text{,} \end{array}$$

(2) $$\begin{array}{c} X_{j}=\left\{X_{j1},X_{j2},X_{jm}\right\}\text{.} \end{array}$$

For the clustering center, if the following is satisfied:

(3) $$\begin{array}{c} d\left(X_{i},W_{e}\right)=\min\;\left\{d\left(X_{i},W_{e}\right),j=1,2,...,k\right\}\text{.} \end{array}$$

Then, the following is considered:

(4) $$\begin{array}{c} X_{i}\in W_{C}\text{.} \end{array}$$

Using the basic idea of combining the statistical method and the data mining algorithm, some existing effective statistical methods are combined with the data mining algorithm to generate some efficient statistical methods and to increase the efficiency of cluster analysis. Similarity measurement method: The clustering analysis algorithm divides the data set into *k* classes, and *k* values can be specified by the user [7]. To achieve the best results, the clustering performance indicator is minimized and allocated to adjacent classes according to the minimum distance [8]. It is quantified by the following distance methods:

(1) Similarity coefficient: it is represented by a number between 0 and 1. If the samples are similar, the value is close to 1; otherwise, it is close to 0.
(2) Distance function: setΩ as sample points, distance function will meet the following formula:
Positive characterization:
  (5) $$\begin{array}{c} D\left(x,y\right)\geq 0\text{.} \end{array}$$
Symmetry:
  (6) $$\begin{array}{c} D\left(x,y\right)=D\left(y,x\right)\text{.} \end{array}$$
Triangle inequality:
  (7) $$\begin{array}{c} D\left(x,y\right)+D\left(y,x\right)\geq D\left(x,z\right)\text{.} \end{array}$$
Or:
  (8) $$\begin{array}{c} D\left(x,y\right)\leq \max\;D\left(x,z\right),D\left(z,y\right)\text{.} \end{array}$$
In the clustering method, the frequently used quantitative methods are as follows:
First, absolute distanceas follows:
  (9) $$\begin{array}{c} D\left(X,Y\right)=\left\{\overset{k}{\underset{i=1}{\sum }}\left|X_{i}-Y_{i}\right|\right\}\text{.} \end{array}$$
Second, Euclidean distance as follows:
  (10) $$\begin{array}{c} D\left(X,Y\right)={\left\{\overset{k}{\underset{i=1}{\sum }}{\left|X_{i}-Y_{i}\right|}^{2}\right\}}^{1/2}\text{.} \end{array}$$
Third, Chebyshev distance as follows:
  (11) $$\begin{array}{c} D\left(X,Y\right)={\left\{\overset{k}{\underset{i=1}{\sum }}{\left|X_{i}-Y_{i}\right|}^{\infty }\right\}}^{1/\infty }\text{.} \end{array}$$
(3) Criterion function:

When the final result of the clustering algorithm satisfies the criterion function, the algorithm ends. In order to improve the accuracy of the clustering algorithm, it is necessary to select the appropriate criterion function [9, 10]. The general criterion functions are as follows:

First, the error square sum criterion function.

Suppose the mixed sample set as follows:

(12) $$\begin{array}{c} X=\left\{x_{1},x_{2},x_{3},...,x_{n}\right\}\text{.} \end{array}$$

In order to measure the instructions of the clustering algorithm, the error sum of the squares criterion function is adopted, and the definition formula is as follows:

(13) $$\begin{array}{c} J_{C}=\overset{C}{\underset{j=1}{\sum }}\overset{n}{\underset{k=1}{\sum }}{\left\|x_{k}^{\left(j\right)}-m_{j}\right\|}^{2}\text{,} \end{array}$$

(14) $$\begin{array}{c} m_{j}=\frac{1}{n_{j}}\left(\overset{n}{\underset{j=1}{\sum }}x_{j}\right)j=1,2,...,c\text{.} \end{array}$$

In the formula, *m*_*j*_ represents the mean value of samples in the jth category and *n*_*j*_ represents the number of samples in the *j*th category [11]. According to the definition of the criterion function in the above formula, it is not difficult to find its value *C* cluster centers and samples in each cluster [12]. The larger the value of *J*_*C*_ is, the larger the clustering error is, and the lower the quality of the clustering algorithm is.

Second, weighted average square distance and criteria are given as follows:

(15) $$\begin{array}{c} J_{I}=\overset{C}{\underset{j=1}{\sum }}P_{j}S_{j}^{*}\text{,} \end{array}$$

(16) $$\begin{array}{c} S_{j}^{*}=\frac{2}{n_{j}\left(n_{j}-1\right)}\underset{x\in x_{i}}{\sum }\underset{x\in x_{j}}{\sum }{\left\|x-x^{\prime }\right\|}^{2}\text{,} \end{array}$$

where *S*_*j*_^*∗*^ is the mean square distance between samples of classes [13]. The weighted average square distance and criterion function can be used to get the correct clustering result.

Third, distance between classes and criteria is as follows:

(17) $$\begin{array}{c} J_{b}=\overset{C}{\underset{j=1}{\sum }}{\left(m_{j}-m\right)}^{2}\text{.} \end{array}$$

In the formula, *m*_*j*_ is the sample mean vector of type *w*_*j*_ and *m* is the mean vector of all samples. The larger the distance between classes and the criterion function, the higher the separation of clustering results and the higher the quality of clustering [14, 15].

## 4. The Language Vowel Recognition System

### 4.1. Speech Recognition System Framework

The speech recognition system is a pattern recognition system in essence, a complete speech recognition system can be roughly divided into the following three parts: (1) speech feature extraction part [16], whose purpose is to extract speech waveform with the change of time speech feature sequence; (2) in the part of the acoustic model and pattern matching, the acoustic model is generated by the acquired speech features through the learning algorithm, and the input simultaneous model of speech features is matched and compared to obtain the recognition results; (3) the language model and language processing. The language model refers to the grammatical network formed by voice recognition commands or the language model formed by statistical methods. The framework of the Mongolian language nonspecific person, large vocabulary and the continuous speech recognition system in this study is shown in Figure 1.

### 4.2. Key Technologies of the Speech Recognition System

#### 4.2.1. Feature Parameter Extraction Technology

Since human vocal organs can only change relatively slowly, speech signals can be approximated as transient and stationary in speech recognition. By dividing the speech signal into data frames of tens of milliseconds, it can be analyzed using various existing digital signal processing techniques [17]. The most commonly used cepstrum feature extraction block diagram is shown in Figure 2.

#### 4.2.2. Selection of Modeling Units

Syllable units are more common in Chinese speech recognition, mainly because Chinese is a monosyllabic language. Although there are about 1300 syllables, there are about 408 atonal voids excluding tone, which is a relatively small number. Phoneme units are often used in the study of English speech recognition. According to the characteristics of Mongolian phonetics and linguistics, we choose phoneme as the lowest modeling unit [18].

#### 4.2.3. Model Training and Pattern Matching Technology

Model training is to obtain model parameters representing the essential characteristics of the model from a large number of known patterns according to certain criteria, while pattern matching is to make the best match between unknown patterns and a model in the model base according to certain criteria. The model training and pattern matching techniques used in speech recognition mainly include dynamic time correction, hidden Markov model, and the artificial neural network.

## 5. Construction of Basic Resources for the Mongolian Continuous Speech Recognition System

### 5.1. Statistical Selection of Corpus

At the word level, there is strong coarticulation between syllables and within syllables. That is, the pronunciation of a vowel or consonant is influenced by its neighboring consonant. The problem of coarticulation cannot be solved by using vowels or consonants alone, which affects the accuracy of speech recognition. Therefore, it is necessary to establish a three-tone model in continuous speech recognition, that is, to consider the influence of the left and right sides of the vowel or consonant adjacent to it. In the selection of language data, we should try to make the selected language data cover all the triphones in Mongolian. In the training of the language model, it is necessary to ensure that each tritone appears no less than 10 times in the corpus to basically ensure the accuracy of the model. When the frequency of occurrence is too small, it is called data sparsity [19].

According to the collected corpus and the characteristics of the Mongolian language, we adopt the method of automatic selection and manual supplement. The word frequency is calculated using the clustering algorithm described above, and the words with greater word frequency are screened out, and these words are considered high-frequency words. Pick out all the sentences that contain the most frequent words and filter out the sentences that are too long and too short. Calculate the priority coefficient; rank each sentence in descending order of priority. Choose some sentences with high priority according to the ranking results. After counting, we selected a corpus of about 16,800 sentences, about 220,000 words, containing more than 10,000 words.

### 5.2. Corpus Construction of the Mongolian Speech Recognition System

Under the guidance of Mongolian corpus construction principles, we have collected about ten thousand words of Mongolian corpus so far. This corpus can be roughly divided into four categories, such as daily language, hotel language, tourism language, textbook, news, and newspapers. Its composition ratio is shown in Table 1.

In order to establish a standard Mongolian sound library, we recorded the students with a relatively standard Mongolian accent. In the process of the language library collection, we mainly follow the following principles:

1. According to the different voice characteristics of men and women, the ratio of male and female recording personnel is 3 : 2
2. Accent must be standard
3. Sound is mature and the waveform is clear

According to the above principles, we collected the voice data of 80 girls and 120 boys. The voice information is stored in the voice database by the recording tool. At the same time, the following information of the recording personnel is also saved in the database: name, gender, age, the native place of the recording personnel, the corpus text read, and so on. The recording tool displays the spoken corpus text sentence-by-sentence to ensure the alignment of the textual corpus with the phonetic corpus [20]. According to the displayed waveform, the quality of speech can be judged and adjusted accordingly.

### 5.3. Construction of Mongolian Speech Recognition System Dictionary

In the establishment of the systematic dictionary, we refer to the domestic and foreign Mongolian language academic circles in the investigation and research of Mongolian dialects commonly used to mark the pronunciation of words. At the same time, considering the simplicity of labeling and the fact that the platform could not recognize some special labeling symbols such as signs, appropriate labeling symbols were adjusted. The final phonetic labeling symbols adopted in the Mongolian speech recognition system dictionary are shown in Tables 2 and 3.

## 6. System Identification Experiment

### 6.1. Identification Experiment

The experiment of this article is to build the acoustic model of the Mongolian continuous speech recognition system based on HTK3.4 and then improve and optimize the HMM model. This article mainly studies the parameter sharing strategy of different models by using the problem set to guide decision tree splitting. Monogol1 (125 Mongolian sentences) and monogol2 (118 Mongolian sentences) were named as the corpus of textbooks for experimental subjects. Dialoguel1 (390 Sentences in Mongolian), dialoguel2 (381 sentences in Mongolian), and dialoguel3 (384 sentences in Mongolian) are divided into three parts [21].

This article makes an experimental comparison between invisible tritones and sparse tritones in the corpus of textbooks and daily dialogues. The experimental process is shown in Figure 3.

#### 6.1.1. Evaluation Criteria of Recognition Results

The evaluation of recognition results is mainly carried out by using the evaluation tool HResults in HTK Toolkit. The resulting results include sentence and word recognition rates and other information. The sentence recognition rate is the ratio of the number of correctly identified sentences to the total number of tested sentences. Word recognition rate graph: Word recognition rate can be obtained by comparing the recognition result word sequence with the reference codex word sequence, which is the correct word-level codex for each sentence.

#### 6.1.2. Experiments on Invisible Tritones

Invisible tritones are those that appear in the test sentence but do not participate in any training process. That is to say, there is no template matching them in the HMM model library participating in the training. The purpose of this experiment is to test the recognition of invisible tritones. Therefore, each part of the textbook corpus and daily conversation corpus are strictly divided into the training corpus and test corpus. On the premise that a certain number of invisible trinosophones appear in the test corpus, the selection of the training corpus should try to ensure that the ratio of male and female corpus reaches 3 : 2.  Table 4 shows the composition of training sentences and test sentences in the experiment.

In our Mongol-all experiment, the number of all tritones generated by the dictionary before the decision number binding is 3373, the number of tritones in the training is 3154, and the number of invisible tritones is 3373–3154 = 219. In the experiment for dialogue-all, the number of all tritones generated by the dictionary before decision number binding is 3185, the number of tritones in the training is 2926, and the number of invisible tritones is 3185–2926 = 259.

During the experiment, we found that the system reported an error when the invisible tritones were identified before the decision tree state binding, and the invisible tritones could not be identified [22]. If invisible tritones are recognized after the decision tree state binding operation, the recognition command can work normally without the system error, and the recognition rate of invisible tritones is certain.  The final results of the experiment are shown in Table 5.

#### 6.1.3. Experiments on Sparse Tritones

Sparse tritones refer to the tritones that occur in training sentences but rarely. Because of the low frequency in the training process, it often cannot get good training. The purpose of this experiment is to test the recognition of sparse tritones before and after the establishment of the decision tree. We divided all the people involved in recording into trainers and testers. The trainer's corpus is used for training, and the tester's corpus is used for identification. The selection of training corpus should ensure that the ratio of male and female corpus should reach 3 : 2.  Table 6 shows the composition of training sentences and test sentences in the experiment [23].

Through experiments, we find that the recognition effect after decision tree state bundling is improved to some extent compared with that before decision tree state bundling. The experimental results before and after decision tree state bundling are shown in Tables 7 and 8.

### 6.2. Identification of Experimental Results

The following conclusions can be drawn from the above experiments:

1. In the experiment of invisible tritones, if invisible tritones are identified without decision tree state binding, the system will report an error. These invisible tritones can be identified effectively after state binding in the decision tree. This is because the invisible tritones to be recognized did not participate in the initial model training process, and the system could not recognize these tritones before the decision tree binding [24].
2. In the experiment of sparse triton, the recognition effect after decision tree state binding is improved to some extent compared with that before decision tree state binding. The maximum improvement percentage of sentence recognition accuracy and word recognition accuracy reached 3.11% and 2.15%, respectively, and the average improvement percentage reached 1.65% and 1.22%, respectively. The comparison of sentence recognition accuracy before and after decision tree state bundling is shown in Figure 4, and the comparison of word recognition accuracy before and after decision tree state bundling is shown in Figure 5.

## 7. Conclusion

In the past, in the study of speech acoustics, the acoustic vowel diagram was only viewed as a fixed vowel diagram or triangular vowel diagram, and the tongue position was described. At present, we find that the theory of the photoacoustic model can better explain that the Mongolian languages are close to each other and have homologous properties after the complete combination of photoacoustic vowel map and photoacoustic pattern map. In summary, the following conclusions can be drawn: (1) Among the relatives of Mongolian languages (Mongolian, Dongxiang, Baoan, Tu, and Eastern Yugu), the vowel acoustic model has the property of linguistic genetic kinship. (2) In addition to the homology of language genesis, there is also the homology of language contact among the relatives of Mongolian languages. (3) By comparing the vowel acoustic models of Mongolian languages, it can be concluded that the vowel acoustic models of the Baoan language, Dongxiang language, and Tu language are the most similar, showing minimal differences and great similarities. Secondly, the acoustical model of Eastern Yugur is not as close as the acoustical model of other relative languages. The acoustical model of Mongolian presents a wider acoustical space than that of other relative languages, almost including other relative languages. We need to combine traditional linguistics and historical linguistics to explain the occurrence of this phenomenon.

Although this article has solved the problem of building the Mongolian phonetic model for speech recognition, there are still many problems to be solved with the continuous expansion and deepening of the research field of speech recognition. In order to make the Mongolian language nonspecific, large vocabulary and the continuous speech recognition system are more perfect. Through experiments, it is found that the experimental results of sparse tritones show that the model has the highest recognition accuracy of 45% for sentences and 86% for words, which is more than 2% higher than before. But in the future, research should be mainly carried out in the following aspects: The establishment of a large vocabulary continuous speech recognition system requires a large corpus. The scale and quality of corpus are two important issues in the construction of corpus. The existing corpus has been strictly screened initially and some bad corpus has been removed. Therefore, some good corpus should be absorbed in the next step to expand the scale of the corpus. In this article, binary grammar and the word network are used as the underlying language model for recognition. Because this language model only considers the correlation between the current word and the previous word, it is not very restrictive to the search space. We should consider using more coherent language models, for example, the ternary model.

## Figures and Tables

**Figure 1:** Speech recognition system framework.

**Figure 2:** Block diagram of MFCC extraction.

**Figure 3:** Experimental process.

**Figure 4:** Comparison of sentence recognition accuracy before and after decision tree binding in sparse triton experiment.

**Figure 5:** Comparison of word recognition accuracy before and after decision tree binding in sparse three-tone subexperiment.

**Table 1:** Composition of the corpus.

Corpus category	Proportion (%)
Everyday language	5
Hotel and tourist expressions	7
Textbook	18
Newspapers	70

**Table 2:** Vowel marks in the dictionary.

Serial number	1	2	3	4	5	6	7
Mongolian letter							
Common sound annotation	a	e	i	o	ud	od	u
Short note annotation	as	es	is	os	uds	ods	us
Long note label	al	el	il	ol	udl	odl	ul

**Table 3:** Marks for prevowels and diphthongs in the dictionary.

Serial number	1	2	3	4	5	6	7	8	9	10
Constituent elements	a + i	a + i	e + i	e + i	o + i	o + i	ud + i	od + i	u + i	u + i
Mark	ae	ael	ee	ei	oe	oel	udi	odi	ui	uil
Serial Number	11	12	13	14	15	16	17	18	19	20
Constituent elements	i + a	i + a	i + ud	u + e	e + u	i + (y) + a	i + (y) + a	i + (y) + e	ud + (w) + a	ud + (w) + a + i
Mark	ia	ial	iud	ue	eu	io	iol	ie	uda	udae

**Table 4:** Composition of training sentences and test sentences in invisible three-tone subexperiment.

Subjects	Number of training sentences	Training the sex ratio	Number of test sentences	Test number of words
Mongol 1	105 *∗* 30 = 3150	1.5	20 *∗* 30 = 600	390 *∗* 30 = 11700
Mongol 2	100 *∗* 30 = 3000	1.5	18 *∗* 30 = 540	240 *∗* 30 = 7200
Mongol-all	6150	1.5	1140	18900
Dialogue 1	325 *∗* 45 = 14625	1.5	65 *∗* 45 = 2925	306 *∗* 45 = 13770
Dialogue 2	318 *∗* 37 = 11766	1.47	63 *∗* 37 = 2331	313 *∗* 37 = 11581
Dialogue 3	320 *∗* 30 = 9600	1.5	64 *∗* 30 = 1920	371 *∗* 30 = 11130
Dialogue-all	35991	1.49	7176	36481

**Table 5:** Invisible triphonon experiment results.

Subjects	Sentence level recognition experimental results				Word level recognition experimental results						
	% Correct	H	S	N	% Correct	ACC	H	D	S	I	N
Mongol 1	9.67	58	542	600	77.67	68.45	9087	342	2271	1078	11700
Mongol 2	18.15	98	442	540	79.54	70.17	5727	137	1336	675	7200
Mongol-all	13.68	156	984	1140	78.38	69.11	14814	479	3607	1753	18900
Dialogue 1	16.03	469	2456	2925	63.55	45.71	8751	351	4668	2457	13770
Dialogue 2	18.66	435	1896	2331	60.33	43.35	6987	289	4305	1967	11581
dialogue 3	13.80	265	1655	1920	59.21	42.90	6590	376	4164	1815	11130
Dialogue-all	16.29	1169	6007	7176	61.20	44.10	22328	1016	13137	6239	36481

**Table 6:** Composition of training sentences and test sentences in sparse three-tone subexperiment.

Subjects	Number of training sentences	Training the sex ratio	Number of test sentences	Test number of words
Mongol 1	125 *∗* 20 = 2500	1.5	125 *∗* 7 = 875	2560 *∗* 7 = 17920
Mongol 2	118 *∗* 22 = 2596	1.44	118 *∗* 6 = 708	1879 *∗* 6 = 11274
Mongol-all	5096	1.47	1583	29194
Dialogue 1	390 *∗* 33 = 12870	1.54	390 *∗* 11 = 4290	1761 *∗* 11 = 19371
Dialogue 2	381 *∗* 27 = 10287	1.45	381 *∗* 9 = 3429	1659 *∗* 9 = 14931
Dialogue 3	384 *∗* 2 = 7680	1.5	384 *∗* 7 = 2688	2001 *∗* 7 = 14007
Dialogue-all	30837	1.5	10407	48309

**Table 7:** Recognition results of decision tree state before extraction.

Subjects	Sentence level recognition experimental results				Word level recognition experimental results						
	% Correct	H	S	N	% Correct	ACC	H	D	S	I	N
Mongol 1	16.34	143	732	875	84.2	78.34	15088	353	2479	1050	17920
Mongol 2	25.14	178	530	708	91.33	84.42	10297	170	807	779	11274
Mongol-all	20.28	321	1262	1583	86.95	80.69	25385	523	3286	1829	29194
Dialogue 1	40.95	1757	2533	4290	83.24	72.96	16124	436	2811	1991	19371
Dialogue 2	43.55	1493	1936	3429	83.04	73.92	12399	292	2240	1362	14931
Dialogue 3	36.57	983	1705	2688	80.66	71.18	11298	278	2431	1328	14007
Dialogue-all	40.67	4233	6174	10407	82.43	72.74	39821	1006	7482	4681	48309

**Table 8:** Recognition results of decision tree state bundling.

Subjects	Sentence level recognition experimental results				Word level recognition experimental results						
	% Correct	H	S	N	% Correct	Acc	H	D	S	I	N
Mongol 1	16.57	145	730	875	84.85	80.49	15206	422	2292	783	17920
Mongol 2	28.25	200	508	708	90.7	86.1	10225	179	870	518	11274
Mongol-all	21.79	345	1238	1583	87.11	82.65	25431	601	3162	1301	29194
Dialogue 1	43.23	1855	2435	4290	83.2	73.74	16117	461	2793	1833	19371
Dialogue 2	44.84	1538	1891	3429	82.71	74.37	12349	293	2289	1245	14931
Dialogue 3	37.95	1020	1668	2688	80.72	71.99	11306	278	2423	1222	14007
Dialogue-all	42.4	4413	5994	10407	82.33	73.43	39772	1032	7505	4300	48309

## Data Availability

The datasets used and analyzed during the current study are available from the corresponding author upon reasonable request.
